# Significance of Magnetic Resonance Imaging Combining with Detection of Serum HE4, TSGF, and CD105 Levels in Diagnosis and Treatment of Moderate to Advanced Cervical Cancer

**DOI:** 10.1155/2022/2090654

**Published:** 2022-02-24

**Authors:** Xiangfu Meng, Yuanmei Qiu, Hongling Wang

**Affiliations:** ^1^Departments of Radiology Linyi Traditional Chinese Medicine Hospital, 211 Jie Fang Road, Linyi, Shandong 276003, China; ^2^Department of Laboratory, South Hospital District of Jiayuguan First People's Hospital, Jiayuguan 735100, Gansu, China; ^3^Department of Clinical Laboratory, Shandong Normal University Hospital, Jinan 250014, Shandong, China

## Abstract

**Objective:**

To explore the significance of magnetic resonance imaging (MRI) combining with detection of serum HE4, TSGF, and CD105 levels in diagnosis and treatment of moderate to advanced cervical cancer.

**Methods:**

By means of retrospective study, 50 patients diagnosed with moderate to advanced cervical cancer by cervix biopsy pathology examination in our hospital from October 2018 to October 2019 were selected as the study group, and another 50 healthy individuals who did not have cervical cancer after routine gynecological examination and conventional ultrasound examination in the same period were selected as the control group. At the time of enrollment and 3 months after treatment, all study subjects received MRI examination and serological examination, and their HE4 and TSGF levels were measured by the enzyme-linked immunosorbent assay (ELISA) and chromatography method, respectively, and additionally, the immunohistochemistry SP method was adopted for patients in the study group to measure the microvessel density (MVD) marked by CD105. The relationship between MRI staging and FIGO staging was assessed, the efficacy of combining MRI with detection of serum HE4, TSGF, and CD105 levels in diagnosing moderate to advanced cervical cancer was calculated by plotting the ROC curve, and the imaging changes and serological changes of tumor tissue before and after treatment were analyzed.

**Results:**

There were 3 of 4 patients in stage IIa and 14 of 15 patients in stage IIIb presenting MRI findings compatible with clinical examinations; 26 patients in stage IIb and 5 patients in stage IVb presenting MRI findings totally compatible with clinical examination. Before treatment, MRI finding of cervical lesion was irregular soft tissue mass, T_1_WI appeared isointensity or hyperintensity, and obvious lesion enhancement could be seen by enhanced scan. T_2_WI appeared mixed signal intensity or hyperintensity, with necrotic tissue and fat suppression being hyperintensity. After treatment, lesions shrunk, originally abnormal signals in 5 patients disappeared, and T_1_WI and T_2_WI signals in 45 patients presented no difference compared to before treatment. After T_1_WI enhancement, mild enhancement could be seen in 41 cases and no enhancement in 4 cases. The CD105-MVD of the study group was (68.98 ± 5.23); before and after treatment, the differences in HE4 and TSGF levels between the study group and the control group were significant (*P* < 0.001). The sensitivity, specificity, and accuracy rate of diagnosis of MRI diagnosis were respectively 82.0% (41/50), 90.0% (45/50), and 86.0% (86/100), and for the diagnosis combining with serum HE4, TSGF, and CD105 levels, they were 96.0% (48/50), 96.0% (48/50), and 96.0% (96/100), respectively, and AUC (95% CI) = 0.960 (0.908–1.000).

**Conclusion:**

MRI staging is objective and accurate and has higher sensitivity when combined with serum HE4, TSGF, and CD105 levels in diagnosing moderate to advanced cervical cancer. All MRI, HE4, and TSGF can reflect the treatment effect of patients and are of great importance to efficacy assessment.

## 1. Introduction

Cervical cancer is a malignant tumor that occurs in the cervix site with nonspecific symptoms at the early stage, and with the development of the disease, patients can present vaginal bleeding, vaginal discharge, and other symptoms. In the late stage, different secondary symptoms will show depending on the extent of cancer foci involvement, such as ureteral obstruction and uremia, and even systemic failure phenomenon such as cachexia in severe cases [1–3]. Although there has been a decreasing trend in the past 40 years [4], the incidence of cervical cancer in China is still increasing. According to a survey report by the World Health Organization in 2018, the incidence and mortality of cervical cancer worldwide is related to the changes in China's social environmental factors as well as the improved diagnostic techniques. Currently, the number of patients who die each year due to cervical cancer in China is above 50,000, accounting for approximately 18.4% of all deaths from female malignancies [5, 6], indicating that the disease is seriously endangering the life health of Chinese women. Performing treatment measures to patients according to clinical stages while actively detecting the treatment effect is key to improving the prognosis of cervical cancer, and in particular, the accuracy of staging in patients with moderate to advanced cervical cancer will directly affect the selection and formulation of treatment options for them. At the present stage, staging of cervical cancer patients is generally performed in practice using the International Federation of Gynaecology and Obstetrics (FIGO) staging method, which provides an important basis for clinical treatment and has the widest application. FIGO is mainly based on pelvic examination, chest radiography, intravenous pyelogram, etc., for diagnosis, in which some of the measures involved belong to invasive examinations, and this staging modality does not incorporate important factors affecting the prognosis of patients, such as tumor volume and lymph node involvement. Therefore, its accuracy remains to be improved [7]. Compared with FIGO, magnetic resonance imaging (MRI) has a better tissue resolution, provides a clearer image of the structural relationship among the cervix, uterus and surrounding tissues and organs, and helps physicians to determine the tumor volume, depth of invasion, and lymph node metastasis, making it a reliable tool to evaluate the clinical stage and treatment effect of patients. Based on the use of MRI, selecting serological markers can improve the diagnostic accuracy rate. HE4 and TSGF are common serological markers in clinic, and a large number of studies have confirmed that HE4 and TSGF are closely associated with the occurrence and progression of cervical cancer [8], so they are important for evaluating the therapeutic effect of cervical cancer patients. CD105 belongs to cell membrane glycoprotein and shows a specific expression status on both tumor tissue and surrounding vascular epidermal cells, and a study by Metcalfe et al. showed that the microvessel density (MVD) marked by CD105 is closely related to the clinical stage and prognosis of cervical cancer patients [9], which may provide a theoretical basis for cervical cancer treatment.

To improve the staging accuracy of patients with moderate to advanced cervical cancer and monitor the treatment effect by low-cost and noninvasive methods at the same time, the study combined MRI and serum HE4, TSGF, and CD105 in the application as follows.

## 2. Materials and Methods

### 2.1. Study Design

It was a retrospective study conducted in our hospital from October 2018 to October 2019, aiming to explore the meaning of MRI combined with detection of serum HE4, TSGF, and CD105 levels in the diagnosis and treatment of moderate to advanced cervical cancer. It was a double-blind study, meaning that neither the research objects nor researchers understood the trial grouping, and the study designer was responsible for arranging and controlling the full trial.

### 2.2. Patient Enrollment

Inclusion criteria were as follows: (1) patients were diagnosed with moderate to advanced cervical cancer after cervix biopsy pathology examination [10]; (2) patients were treated in our hospital in the whole course and did not transfer to other hospitals before completion of the study; (3) the estimated survival of the patients was over 3 months; (4) patients had good liver and kidney functions; (5) patients were at least 18 years old; (6) patients' score on physical status was less than 2 points; (7) the diameter of tumor was between 4 and 10 cm; and (8) patients met surgical indication. Exclusion criteria were as follows: (1) patients could not communicate with others due to factors including hearing disorder, language disorder, unconsciousness, and mental diseases; (2) pregnant or lactating women; (3) patients had other severe organic diseases; (4) patients could not go along with sampling; and (5) patients had radiotherapy or surgical contraindications.

### 2.3. Grouping of Study Subjects

According to the inclusion and exclusion criteria, 50 patients diagnosed with moderate to advanced cervical cancer by cervix biopsy pathology examination in our hospital from October 2018 to October 2019 were selected as the study group, and another 50 healthy individuals who did not have cervical cancer after routine gynecological examination and conventional ultrasound examination in the same period were selected as the control group. Between the study group and the control group, no statistical differences in patients' general data such as mean age (51.46 ± 14.22 vs. 51.44 ± 14.26 years), mean body mass (58.65 ± 2.65 vs. 58.70 ± 2.54 kg), and mean BMI (21.45 ± 1.66 vs. 21.55 ± 1.58 kg/m^2^) were observed (*P* > 0.05). In the study group, there were 18 cases with cystadenocarcinoma, 20 cases with squamous cell carcinoma, and 12 cases with adenosquamous carcinoma, and all patients were treated with surgery combined with radiotherapy.

### 2.4. Moral Consideration

The study met the principles of the *World Medical Association Declaration of Helsinki (2013)* [11], and patients and their family members signed the informed consent.

### 2.5. Methods

#### 2.5.1. Imaging Examination

At the time of enrollment and 3 months after treatment, all study subjects received MRI examination, for some patients placed with the metal contraceptive ring in their uterine cavity, the ring was removed before examination. After fasting for 5 days, patients drank enough water to fill the bladder (overfilling should be avoided), received scan in the supine position with the head coming in first, during which the patients breathed lightly and held both arms above the top of the head, and the scan was performed from their pubic symphysis to superior iliac spine. The patients' MRI examination findings were determined by 2 senior clinical physicians jointly reading the slides. The GE Singa Excite 3.0 T MRI scanner (NAPA registration (I) no. 20153333982) and body matrix coil were selected to perform pelvic MRI plain scan and enhanced scan, with FOV = 350–400 mm, matrix 256×256, and reconstruction matrix 512×512. (1) Plain scan: SE T_1_WI, TR = 300–500 ms, TE = 10–20 ms, and the number of excitation was 4; TSE T_2_WI, TR = 2,000–2,500 ms, TE = 120 ms, and the number of excitation was 6; TSE T_2_WI plus short TI inversion recovery (STIR), TR = 2,000–2,500 ms, TE = 100 ms, and the number of excitation was 4–6; echo chain 15–25. (2) Enhanced scan: after intravenous injection of 0.01 mmol/kg of contrast agent gadopentetate dimeglumine (Beijing Beilu Pharmaceutical Co., Ltd.; NMPA approval no. H10860002), SE T_1_WI-enhanced axial and sagittal scans were performed.

#### 2.5.2. Serological Examination

At the time of enrollment and 3 months after treatment, all study subjects received the serological examination. In one morning of patients' nonmenstrual period, 5 ml of fasting venous blood was drawn and placed in a centrifugal tube not containing anticoagulant for the detection of HE4 and TSGF levels, respectively, by the ELISA method (Beijing Kewei Clinical Diagnostic Reagent Inc.; NMPA approval no. S20060028) and chromatography method (ACON Biotech (Hangzhou) Co., Ltd., original matched kits; Zhejiang MPA certified no. 20122400529).

#### 2.5.3. CD105

The cancer tissues removed from the patients in the study group during surgery were subjected to routine preparation, and the immunohistochemistry SP method (Beijing Kewei Clinical Diagnostic Reagent Inc., NMPA approval no. S20060028) was performed. To be specific, the tissue sections were deparaffinized by xylene, dehydrated by gradient ethanol, and subjected to immunohistochemical staining, DAB coloration, hematoxylin counterstaining, neutral gum mounting, and microscopic observation according to the steps in the specification. PBS was substituted for the primary antibody as a negative control, and mouse anti-human CD105 monoclonal antibody (clone Sn6h, dilution 1 : 2) was a Dako product.

### 2.6. Observation Criteria

#### 2.6.1. Patients' Clinical Stages

Before treatment, FIGO staging (2009) [12] and MRI staging [13] were adopted for patients, and the results from the two staging methods were recorded.

#### 2.6.2. MRI Imaging Characteristics

By comparing with the imaging characteristics of normal cervix MRI, the lesions were classified into isointensity, slightly hyperintensity, and hyperintensity so as to analyze the MRI imaging characteristics of patients with moderate to advanced cervical cancer 3 months before and after treatment. Criterion for treatment effect: it was regarded as significantly effective if the signal of the tumor tissue changed to normal after the end of treatment or appeared isointensity or hypointensity on T_2_WI and “no enhancement zone” appeared in enhanced T_1_WI.

#### 2.6.3. HE4, TSGF, and CD105 Levels

The HE4 and TSGF levels of patients in the study group 3 months before and after treatment were compared, and the situation of CD105-MVD was recorded. According to the Weidner method [14], the area that stained brownish yellow was taken as the blood vessel, the sections were first observed under low magnification (40×) comprehensively to determine where the density of blood vessels within the tumor was highest and then examined at high magnification (400×) to count the number of microvessels of 3 fields, and its average value was taken as the MVD value.

### 2.7. Statistical Processing

In this study, the data processing software was SPSS20.0, the picture drawing software was GraphPad Prism 7 (GraphPad Software, San Diego, USA), the items included were enumeration data and measurement data, the methods used were the *χ*^2^ test and *t*-test, and differences were considered statistically significant at *P* < 0.05.

## 3. Results

### 3.1. Patients' Clinical Stages

Among 4 patients in stage IIa, 3 patients presented MRI findings compatible with clinical examination, and 1 patient was in stage IIb by MRI. Among 15 patients in stage IIIb, 14 patients presented MRI findings compatible with clinical examination, and 1 patient showed ischium metastasis and was in stage IVb by MRI. 26 patients in stage IIb and 5 patients in stage IVb presented MRI findings completely compatible with clinical examination (see Table 1).

### 3.2. MRI Imaging Characteristics

Before treatment, MRI finding of the cervical lesion was irregular soft tissue mass, T_1_WI appeared isointensity or hyperintensity, and obvious lesion enhancement could be seen by enhanced scan. T_2_WI appeared mixed signal intensity or hyperintensity, with necrotic tissue and fat suppression being hyperintensity. Pelvic lymph node metastasis T_1_WI presented hyperintensity, obvious focus enhancement could be seen by enhanced scan, and T_2_WI presented mixed signal intensity; see Figure 1 for classic cases. Through the examination conducted 3 months after treatment, it was found that lesions shrunk, originally abnormal signals in 5 patients disappeared, T_1_WI and T_2_WI signals in 45 patients presented no difference compared to before treatment, and after T_1_WI enhancement, mild enhancement could be seen in 41 cases and no enhancement in 4 cases (see Figure 2).

### 3.3. HE4, TSGF, and CD105 Levels

The CD105-MVD of the study group was (68.98 ± 5.23); before and after treatment, HE4 and TSGF levels were significantly different between the study group and the control group (*P* < 0.001) (see Figure 3).

The HE4 levels of the study group before and after treatment were (192.65 ± 9.67) pmol/L and (145.68 ± 8.55) pmol/L, respectively, and the HE4 level of the control group was (65.84 ± 4.22) pmol/L.

The TSGF levels of the study group before and after treatment were (90.65 ± 5.22) U/ml and (76.55 ± 6.32) U/ml, respectively, and the TSGF level of the control group was (45.32 ± 3.68) U/ml.

### 3.4. ROC Curve

The sensitivity, specificity, and accuracy rate of diagnosis of MRI diagnosis were respectively 82.0% (41/50), 90.0% (45/50), and 86.0% (86/100), and for the diagnosis combined with serum HE4, TSGF, and CD105, they were 96.0% (48/50), 96.0% (48/50), and 96.0% (96/100), respectively, and AUC (95% CI) = 0.960 (0.908–1.000) (see Figure 4).

## 4. Discussion

Cervical cancer is a common malignancy of the female reproductive system, and epidemiological data in 2014 showed that the incidence of cervical cancer in urban and rural areas of China still presented an increasing trend (49,600/100,000 and 23,900/100,000 in 1989–1990 to 119,800/100,000 and 117,700/100,000 in 2007–2008), and more and more younger patients suffered from the disease [15], so further relevant studies on diagnostic measures for cervical cancer need to be strengthened. At present, the diagnosis of cervical cancer mainly depends on gynecological examination and cytology examination, and in clinic, the disease stage is usually determined based on FIGO. However, the precision of FIGO is subject to the experience and subjective judgment of examiners, so it has limitations in diagnosing the stage of lesions, and incorrect estimation of the extent of tumor invasion often occurs in practice [16], which affects the selection of treatment options. Treatment options are crucial elements affecting the prognosis of cervical cancer patients, especially for those in the middle and advanced stages. Treatment measures must be developed based on accurate clinical staging, and surgical treatment is not advisable for patients with the presence of parametrial and vaginal involvement, so comprehensive therapeutic measures based on radiation therapy are required [17]. Therefore, it is of great importance to the choice of a more objective diagnostic modality. Currently, MRI is widely used in practice because of its advantages including high tissue resolution, multiple sequences, and multiparametric imaging; its T_1_WI sequence allows visualization of lesion invasion in parametrial adipose tissue; and its T_2_WI sequence enables visualization of tumor parametrial and vaginal invasion. The study by scholars Ahmed Hiba Z et al. showed that the accuracy of MRI in evaluating parametrial and vaginal invasion was 94% and 81%, respectively [18], while STIR sequence can be used to exclude the interference factors of fat signal and further improve the accuracy of T_2_WI sequence. T_2_WI is the primary imaging sequence for MRI staging of cervical cancer, and this study showed that a total of 48 patients presented MRI findings completely compatible with clinical examination, indicating that there was a definite efficacy of MRI in diagnosing clinical stages of cervical cancer.

In addition, MRI also works well in the treatment of cervical cancer. Radiotherapy is generally administered to patients with moderate to advanced cervical cancer, and some patients also undergo comprehensive treatment consisting of surgery. Overall, assessment of tumor sensitivity to radiotherapy is key to selecting treatment options. Gynecological examination is less clinically useful than MRI because it is subjective and does not precisely assess the necrosis and residual status of the tumor. MRI has the advantages such as zero radiation and easy operation, which can objectively evaluate the progression and regression of lesions, and in particular, T_1_WI-enhanced scan can show the ischemic and necrotic areas within the tumor at an early stage, which is beneficial for predicting the effect of radiotherapy [19–21]. The study found that before treatment, MRI finding of cervical lesion was irregular soft tissue mass, T_2_WI appeared mixed signal intensity or hyperintensity, with necrotic tissue and fat suppression being hyperintensity; after treatment, lesions shrunk, originally abnormal signals in 5 patients disappeared, and after T_1_WI enhancement, mild enhancement could be seen in 41 patients and no enhancement in 4 patients, which demonstrated that MRI could provide more valuable information of efficacy assessment for the clinical physicians. Moreover, patients' HE4 and TSGF levels reduced after treatment, proving that such indicators could dynamically assess patients' prognosis. Both HE4 and TSGF are clinically common markers for diagnosing cervical cancer, respectively, with an accuracy rate of up to 80.0% and 64.5%–71.8% [22]. Scholars Su et al. reported that TSGF also has some merits in determining cervical cancer stage and is highly correlative with clinicopathological characteristics of cervical cancer, with *γ* = 0.416 and *P* < 0.01 [23]. As a cell membrane glycoprotein closely related to neovascularization, its MVD value is also associated with cervical cancer stage and lymph node metastasis [24, 25]. This study did not explore the relationship among TSGF, CD105-MVD, and cervical cancer staging, but the efficacy difference between MRI diagnosis and MRI combined with HE4, TSGF, and CD105 diagnosis of advanced cervical cancer was compared, and it was found that the combined diagnosis had an accuracy rate of 96.0% (96/100), AUC (95% CI) = 0.960 (0.908–1.000), which confirmed that combining the four presented an ideal diagnostic efficacy. The expression levels of HE4, TSGF, and CD105-MVD in different clinical stages of cervical cancer need to be further explored to provide new ideas for targeted drug therapy of moderate to advanced cervical cancer.

In conclusion, MRI staging is objective and correct, presents high sensitivity in diagnosing cervical cancer when combined with serum HE4, TSGF, and CD105 levels, and can evaluate patients' clinical staging. All MRI, HE4, and TSGF can reflect the treatment effect of patients and are of great significance to assess the efficacy of patients.

## Figures and Tables

**Figure 1:** Patients with cervical squamous adenocarcinoma with MRI findings completely compatible with clinical examination.

**Figure 2:** MRI findings of patients with cervical adenocarcinoma after 3 months of treatment.

**Figure 3:** HE4 and TSGF levels (*x* ± *s*). # indicated *P* < 0.001.

**Figure 4:** Diagnosis efficacy analysis of different diagnosis methods.

**Table 1:** Comparison of FIGO staging and MRI staging.

Method	IIa	IIb	IIIb	IVb
FIGO staging	4 (8.0)	26 (52.0)	15 (30.0)	5 (10.0)
MRI staging	3 (6.0)	27 (54.0)	14 (28.0)	6 (12.0)

## Data Availability

The data to support the findings of this study are available on reasonable request from the corresponding author.
